The article "Model Selection and Identification of Osteoporosis Risk Factors in Women to Improve Their Healthcare" was published in 2023. Journal: J Healthc Eng.

# Model Selection and Identification of Osteoporosis Risk Factors in Women to Improve Their Healthcare

**DOI:** 10.1155/2023/3571769

**Published:** 2023-07-04

**Authors:** Faisal Maqbool Zahid, Shahla Faisal, Shahid Kamal, Khawar Shahzad, Seemi Iram, Bright Opoku Ahinkorah, Abdul-Aziz Seidu, Abid Rasheed, John Elvis Hagan

**Affiliations:** ^1^Department of Statistics, Government College University, Faisalabad, Pakistan; ^2^Center of Data Science, Government College University, Faisalabad, Pakistan; ^3^College of Statistical and Actuarial Sciences, University of the Punjab, Lahore, Pakistan; ^4^Consultant Orthopedic Surgeon, District Headquarters (DHQ) Hospital, Faisalabad, Pakistan; ^5^School of Public Health, University of Technology Sydney, Sydney, New South Wales 2007, Australia; ^6^Department of Estate Management, Takoradi Technical University, Takoradi, Ghana; ^7^Centre for Gender and Advocacy, Takoradi Technical University, Takoradi, Ghana; ^8^College of Public Health, Medical and Veterinary Sciences, James Cook University, Townsville, Queensland 4811, Australia; ^9^Faculty of Medical Sciences, Government College University, Faisalabad, Pakistan; ^10^Department of Health, Physical Education,and Recreation, University of Cape Coast, Cape Coast, PMB, Ghana; ^11^Neurocognition and Action-Biomechanics-Research Group, Faculty of Psychology and Sports Science, Bielefeld University, Postfach 10 01 31, 33501 Bielefeld, Germany

## Abstract

Osteoporosis is characterized by low bone mineral density leading to enhanced bone fragility and a consequent increase in fracture risk. The focus of this case-control study was to identify significant socioeconomic risk factors of osteoporosis in Pakistani women and examine how the risk increases for different levels of risk factors. A case-control study was conducted from November 2018 to August 2019 in two main hospitals in Faisalabad, Pakistan. Multiple logistic regression was used to explore the significant risk factors of osteoporosis and how the risk increases in cases (cases = 120) as compared to the control group (controls = 120) in the presence of these risk factors. The mean age ± standard deviation for cases and controls was 59.62 ± 10.75 and 54.27 ± 10.09, respectively. The minimum and maximum ages were 36 and 80 years, respectively. In addition to age, bone fracture, family history, regular physical activity, family size, use of meat, type of birth, breastfeeding, premature menopause, loss of appetite, and use of anticoagulants were significant risk factors with *p*-values less than 0.05. The risk prediction model with significant risk factors was a good fit with a *p*-value of 0.28, corresponding to the Hosmer–Lemeshow test value (*χ*2 = 9.78). This parsimonious model with Cox–Snell *R*2 = 0.50 (with a maximum value = 0.75) and Nagelkerke *R*2 = 0.66 showed an AUC of 0.924 as compared to the full model with all risk factors under study that exhibited an AUC of 0.949.

## 1. Introduction

Osteoporosis is not only the prime root of fractures, but it also files a high rank among abnormalities that cause people dependent and bedridden with serious issues [1]. According to an estimate of the WHO [1], osteoporosis causes more than 8.9 million fractures annually worldwide. The estimated number of fractures in Pakistan due to osteoporosis is 9.91 million (7.19 million in women and 2.71 million in men), which is expected to rise to 11.3 million in 2020 and 12.91 million in 2050 [2]. In the last twenty years, the life expectancy at birth in Pakistan has increased by 5.5 years, which is also the reason for the increase in the population suffering from osteoporosis [3, 4]. Osteoporosis is a silent disease, and there are often no symptoms until the first fracture occurs [5]. Fracture is the most significant health issue of osteoporosis. Bones with normal bone mass have a dense matrix of bone cells, whereas osteoporotic bone dissolves and is left with thin strands, resulting in an increase in bone fragility and leading to fracture [6].

Osteoporotic fractures are the leading cause of morbidity and mortality after being discharged from a hospital [1]. The main osteoporosis fractures are hip, forearm, wrist, spine, and proximal humerus fractures [1]. The osteoporotic fractures are expected to touch a figure of 11.3 million in 2020 and 12.91 million in 2050 [7]. According to Sözen et al. [8], osteoporotic fractures not only cause 15–20% increase death rates per year but also cause social segregation, recession, and require long-term care. The age-specific hip fractures in men are half than those in women in most communities [5].

Most of the studies uncover that the process of osteoporosis hastes after menopause in women due to low estrogen levels [9–11]. According to Thulkar and Singh [9], the rate of bone loss due to menopause is 2–5% per year. Different studies revealed that older age is a prime factor of fragile bone [11, 12]. Females are more prone to osteoporotic fractures than are males worldwide [13]. Females with a positive family history of osteoporosis and those who are using steroids or medications for chronic diseases are more exposed to the disease. However, the use of calcium supplements and hormone replacement therapy can be taken as preventive and protective measures [14]. Barret-Connor et al. [15] reported low bone mineral density (BMD) among Asian women compared to other ethnic groups around the globe. Mithal and Kaur [7] predicted that, by 2050, half of the global osteoporotic fractures will be in the Asian population. In consonance with various epidemiological predictions, until 2050, over 70% of all osteoporotic fractures will occur in specific regions of the world including Asia, the Middle East, and Latin America [16]. According to [17, 18], for every osteoporotic man, four women are suffering from osteoporosis. According to Hafeez et al. [13], women from the Indian subcontinent are at a high risk of facing osteoporosis compared to the Caucasian race.

Osteoporosis has not been taken seriously in developing countries, especially in Pakistan. In Asia generally, and in Pakistan specifically, there is a lack of medical facilities and equipment to diagnose osteoporosis and its treatment. The rural population of Pakistan has very little knowledge about dietetics and bone density [10]. In a study in the most populated city, i.e., Karachi of Pakistan, Habib et al. [19] reported a 16.4% prevalence of the disease. It is a dilemma that statistics about the prevalence of osteoporosis and osteoporotic fractures are scarce in Pakistan [13, 19, 20]. Even this disease has not been taken seriously by a common person due to many reasons, e.g., poor literacy rates, lack of awareness about the disease and nutritional imbalance, and considering osteoporosis as the disease of old age and developed states [7, 19, 21]. There is no database or statistics available at the government level about this disease. For research, we are still relying on the western literature about osteoporosis and its diagnosis, cutoff values, and associated risk factors. In addition, rare Pakistani studies are available in the literature that are based on primary data collected from some small-scale studies. Faisalabad is the third largest and the most populated and major industrial city of Pakistan. To the best of our knowledge, no study is available in this region to investigate the prevalence of osteoporosis and the risk factors associated with it. This study is an effort to fill this gap. The main intent of this paper is to identify significant socioeconomic risk factors of osteoporosis in Pakistani women and examine how the risk increases for different levels of risk factors in females of age groups of 30 years or more.

## 2. Materials and Methods

### 2.1. Study Area

Faisalabad is a major industrial city of Pakistan located in the center of the most populous province of Pakistan, i.e., Punjab. It is the third biggest city in Pakistan with respect to size and population. The study was conducted in the two main teaching hospitals of Faisalabad, i.e., District Head Quarter (DHQ) Hospital and Allied Hospital.

### 2.2. Study Design

The study was a case-control study with a 1 : 1 case-control ratio, and convenient sampling was considered to collect the information from cases and controls.

### 2.3. Duration of the Study and Data

The case-control study was completed in the two teaching hospitals; District Head Quarter (DHQ) Hospital and Allied Hospital, Faisalabad. These two hospitals not only cover the population of Faisalabad city but also manage the patients of the whole Faisalabad division due to the available medical facilities. The study was completed from October 2018–August 2019.

### 2.4. Inclusion Criteria

Females of age ≥30 years were considered for the study. We considered this age because peak bone mass occurs around the age of 30 years and reduction starts from 40 years of age [22]. Osteoporotic patients were decided based on digital X-ray radiogrammetry. Females having a Metacarpal Index (MCI) value less than 0.4 were considered osteoporotic, whereas an index value higher than 0.6 was considered for the control group [23].

### 2.5. Sampling Technique and Sample Size

Nagi et al. [24] reported that there are 9.9 million people in Pakistan who are osteoporosis sufferers, among which 7.2 million are women. We used the WHO calculator [25] to obtain the sample size. The estimated sample size with a 95% confidence interval and a 6% margin of error was 240 with a 1 : 1 case-control ratio. We used the convenience sampling technique to select 120 cases, i.e., premenopausal and postmenopausal females with age ≥30 years who were suffering from osteoporosis and 120 controls, i.e., females who were not osteoporosis sufferers.

### 2.6. Risk Factors

In the literature, different researchers have used different risk factors in their studies [2, 6, 10–16, 19–21]. We tried to consider all of them to investigate how each risk factor increases the risk in osteoporotic females compared to nonsufferers in the presence of other factors. The information about different demographic and socioeconomic risk factors was collected through structured questionnaires with the prior consent of the subjects. Information about the following possible risk factors was collected: age, BMI, locality, education, awareness about the disease, regular physical activity, exposure to sunlight, reproductive history, gynaecological status, and loss of weight. Others were intake of calcium through natural sources and supplements, use of proteins, history of fracture, family history of osteoporosis, number and kind of births, monthly household income, ownership of the house, and use of anticoagulants.

### 2.7. Ethical Issues

The study was conducted after the approval of the Ethical Review Committee of Govt. College University Faisalabad. The same approval was taken from both hospitals where the study was conducted. The respondents were informed about the study and its objectives before their interview. After knowing about the study, the respondents who agreed to be a part of the study were included in the research.

### 2.8. Statistical Techniques

Both descriptive and inferential analyses were employed in this study. The inferential analyses were used in drawing the significance of risk factors and the selection of a risk prediction model. Descriptive statistics were considered for continuous demographic and socioeconomic risk factors in terms of mean and standard deviation, whereas frequencies and percentages were considered for qualitative factors. To explore significant risk factors, a logistic regression model was fitted for a dichotomous response mentioning whether a subject is osteoporotic or not. The odds ratios and their confidence intervals were computed for comparing the relative odds of osteoporosis in the presence of a given risk factor. The multiple logistic regression model with *p* risk factors (predictors) X_1_, X_2_,…, X_*p*_, without interaction terms, is defined as

(1) $$\begin{array}{c} logit\left[\pi \left(x\right)\right]=\log\left[\frac{\pi \left(x\right)}{1-\pi \left(x\right)}\right]=\beta_{0}+\beta_{1}X_{1}+\ldots +\beta_{p}X_{p}\text{,} \end{array}$$

where *β*'s are the regression coefficients of predictors. The statistical programming language *R* was used to fit the logistic regression model, test the significance of parameter estimates, and compute the odds ratios and their corresponding confidence intervals. The significance of parameter estimates associated with different risk factors was tested using the Wald test. The goodness of fit for the risk prediction model was confirmed using the Hosmer–Lemeshow test [26]. Additionally, Cox–Snell R^2^ [27] and its adjusted version, that is, Nagelkerke R^2^ [28], were computed to study the variation in the response variable explained by the model. The usual R^2^ in case of linear regression is also a special case of Cox–Snell R^2^. Usual R^2^ has a maximum value of 1, but for Cox–Snell R^2^, it is less than one. However, Nagelkerke R^2^ has an upper bound of 1 just like the case with linear models.

## 3. Results

Our focus was on females with age ≥30 because they are more exposed to this disease than males [13, 17, 18]. The average age of the whole sample was 56.95 years (54.27 years for cases and 59.62 years for the control group) with a standard deviation of 10.74 years (6.64 and 5.78 years for cases and controls, respectively). The mean ± SD of the family size was 6.68 ± 2.62 and 6.87 ± 3.45 for the control and patient groups, respectively. The average BMI (body mass index) was little higher in cases (30.95) than in controls (28.10), whereas the average age at menarche was almost the same in both groups, with an average of 14.25 years in the whole sample (Table 1).

The percentage of literate patients and those who have awareness about the disease was low, i.e., 25% and 5%, respectively. The incidence of bone fracture is 35% higher in cases than that in the control group. Among the osteoporotic females considered in our study, 43 were admitted to the hospital for hip fracture surgery, 16 for tibial fracture, and four for some other fracture surgery. Fifty-seven cases had no fracture. In the control group, one woman was admitted to the hospital for hip fracture surgery, six for tibial fracture, fourteen for some other fracture surgery, and 99 had no fracture. Only 13% of cases had a family history of the disease. Fewer patients (14%) were observed to be involved in regular physical activity compared to nonsufferers (64%). The percentage of patients who do not drink milk at least once a week is 19% more than that in the control group. The frequency of eating meat at least once a week was 21% higher in the control group than that in the patient group. In our sample, more than 80% of women had natural delivery in cases and controls as well. There are 90% of women in both groups who fed their children before suffering from the disease. Normal menopause, normal menstrual flow, and 4–7 days of a menstrual cycle were observed in most women in both groups. Most women were not using any calcium supplements. Compared to healthy women (26%), a high percentage (80%) of females suffering from osteoporosis complained of the loss of weight. Half of the patients reported poor appetite (Table 1).

The significant risk factors were age, bone fracture, family history of the disease, daily physical activity, number of family members living in a house, frequency of eating meat, kind of delivery, breastfeeding, menopausal status, appetite, and use of anticoagulants. The results showed that a one-year increase in age may cause a 10% increase in the odds of being osteoporotic. In the case of bone fractures, the odds of disease are 3.5 times higher than those who have not got a fracture. Chances increase 36 times to be a patient of osteoporosis in the case of having a history in the family. The number of persons living in a house is also identified as a significant risk factor, with 24% higher odds for an increase of one member in the same size of the house. The occasional use of meat was not found to be a significant risk factor, but the frequent use of meat (at least once a week) decreases the chances of osteoporosis. The person who eats meat at least once a week is 76% safer than that person who is the occasional consumer of meat. Since the duration of breastfeeding is correlated with the number of births, the results showed that an increased number of births and consequently breastfeeding increase the risk a lot. According to our study, a woman who has fed in the past is seven times more exposed to the disease. The risk in the mothers who were feeding during our study, i.e., feeding as a patient, possessed 120 times more risk than those females who did not feed as a patient. Abnormal menopause in females may also increase the risk of osteoporosis eight times. The results of the study reflected that the chances of suffering from the disease are 91% higher in females who have an issue of loss of appetite. Anticoagulants users are also observed twenty times more exposed to the disease than nonusers. The parameter estimates, their standard errors, Wald-test statistic value, odds ratio, and its 95% confidence interval are given in Table 2. A risk prediction model with significant risk factors was fitted, and the goodness of fit of that model was tested with the Hosmer–Lemeshow test [26]. The test showed that the fitted model is a good fit with a *p* value of 0.28 for the test-statistic value of *χ*2 = 9.78. The values of different pseudo-R^2^ were computed for different possible models with available risk factors. The model with significant risk factors showed Cox–Snell's R^2^ [27] value of 0.50 corresponding to a maximum value of 0.75. Another pseudo measure of R^2^ is Nagelkerke/Crag and Uhler's R^2^ [28], which is an adjusted version of Cox–Snell R^2^ with a maximum value of 1. This pseudo measure resulted in a value of 0.66. 

These measures were better than all possible models fitted with the risk factors under study except the model with all risk factors. These measures were better than all possible models fitted with the risk factors under study except the model with all risk factors. Although the model with all risk factors showed little improvement in the pseudo-R^2^ values (Cox–Snell *R*2 = 0.55 and Nagelkerke *R*2 = 0.73), but at the same time, most of the factors in this model were insignificant.

The ROC curve (receiver operating characteristic curve) describing the trade-off between sensitivity (true positive rate) and 1-specificity (false positive rate) for the models with all risk factors and significant risk factors is shown in Figure 1. Both curves show that the performance of a parsimonious model with significant risk factors is as good as for the overall model. The area under the curve (AUC) is approximately the same for both models. The calibration curve in Figure 1 also reflects that a parsimonious model with significant risk factors can be a good choice as an alternative to a rich model with a large number of possible risk factors.

## 4. Discussion

In our study, prevalence of osteoporosis was observed to increase with growing age, especially starting from the age of 40 years, which is in accordance with different other studies [29–31]. Age was found to be a significant factor causing osteoporosis similar to the findings in [12, 14, 16, 19, 24, 32–34]. However, according to [35], age was not a significant factor causing osteoporosis. The BMI did not show a significant effect in predicting osteoporosis in our study. The BMI was also not significant in other studies, where height and weight were significant at the same time [12, 13, 32, 36, 37]. In a systematic evaluation, the authors of [38] explored that birth weight has a negative association with BMD and a positive association with fracture risk. A family history of osteoporosis and malnourishment has also been found to be the cause of low BMD [39]. The history of fractures can be helpful to identify the presence of osteoporosis, as identified by [2, 40]. The results of [41, 42] about the significance of exercise/involvement in physical activities match our findings. The number of parity that we considered in this study as the family size also appeared as a significant risk factor [16, 32, 34, 40]. We found that, with an increasing number in parity, the risk of osteoporosis also increases. Also, the kind of delivery that is normal or operated, as compared to those females who had zero parity or gravidity, has an impact on the risk of osteoporosis. Different studies [16, 32, 41] are available in the support of our finding that breastfeeding also significantly increases the risk of osteoporosis. According to our investigation, low appetite can also be a significant factor for identifying the osteoporosis patient. The use of anticoagulants may also significantly increase the risk of osteoporosis. Naz et al. [32] found that diabetes can increase the risk of being osteoporotic, but in our study, comorbidity was not a significant risk factor. Our finding about the significance of abnormal menopause was also consistent with other studies [2, 16, 40]. Fatima et al. [40] in their research found the ownership of the house as a significant risk factor, but in our study, neither this factor nor the income level was found to be a significant risk factor. In some studies [33, 41], the use of calcium supplements has been found to be a significant factor, but in our study, this was not the case.

## 5. Conclusion

This study was an attempt to address the neglected medical problem of osteoporosis in females and the risk factors associated with it in Pakistan. To cope with this growing issue, we need (i) diagnostic facilities, e.g., DEXA scan or QUS, i.e., quantitative ultrasound, (ii) population-based studies at the government level and some health programs at the national level focusing on this disease, and (iii) awareness and education among people about osteoporosis, its diagnosis, treatment, and adoption of possible changed lifestyles for this disease.

## Figures and Tables

**Figure 1:** ROC curve (a) and calibration curves (b) for the overall model and parsimonious model with significant risk factors.

**Table 1:** Frequencies and percentages of categorical risk factors.

Variable	Categories	Control	% age	Case	% age	Variable	Categories	Control	% age	Case	% age
Locality	Urban	59	49.17	65	54.17	Delivery kind	None	5	4.17	10	8.33
	Rural	61	50.83	55	45.83		Normal	104	86.67	100	83.33
Literacy	Illiterate	73	60.83	90	75		Major	11	9.17	10	8.33
	Literate	47	39.17	30	25	Feeding as a mother	No	13	10.83	12	10
Awareness	No	108	90	114	95		Yes	107	89.17	108	90
	Yes	12	10	6	5	Feeding as a patient	No	9	7.5	2	1.67
Symptoms	Tiredness	29	24.17	41	34.17		Yes	111	92.5	118	98.33
	Body pain	91	75.83	79	65.83	Menopause status	Normal	106	88.33	94	78.33
Fracture	No	99	82.5	57	47.5		Abnormal	14	11.67	26	21.67
	Yes	21	17.5	63	52.5	Menstruation frequency	High	20	16.67	28	23.33
Fracture history	No	110	91.67	92	76.67		Normal	100	83.33	92	76.67
	Yes	10	8.33	28	23.33	Menstruation duration	4–7 days	117	97.5	110	91.67
Family history	No	117	97.5	104	86.67		≥8 days	3	2.5	10	8.33
	Yes	3	2.5	16	13.33	Menstruation regularity	Irregular	2	1.67	6	5
Physical activity	No	43	35.83	103	85.83		Regular	118	98.33	114	95
	Yes	77	64.17	17	14.17	Regular calcium intake	No	100	83.33	106	88.33
Sun exposure	No	22	18.33	38	31.67		Yes	20	16.67	14	11.67
	Yes	98	81.67	82	68.33	Appetite	Poor	17	14.17	58	48.33
Calcium in preg	No	100	83.33	111	92.5		Normal	103	85.83	62	51.67
	Yes	20	16.67	9	7.5	Abdomen system	Abnormal	23	19.17	56	46.67
House owned	Rented	14	11.67	16	13.33		Normal	97	80.83	64	53.33
	Owned	106	88.33	104	86.67	Sleep disturbance	No	91	75.83	42	35
Milk	0	56	46.67	78	65		Yes	29	24.17	78	65
	>=1	64	53.33	42	35	Mental stress	No	101	84.17	55	45.83
Meat	None	8	6.67	20	16.67		Yes	19	15.83	65	54.17
	Red	30	25	21	17.5	Comorbidity	No	93	77.5	26	21.67
	White + red	82	68.33	79	65.83		Yes	27	22.5	94	78.33
Meat frequency	0	47	39.17	73	60.83	Anticoagulants	No	118	98.33	102	85
	>=1	73	60.83	47	39.17		Yes	2	1.67	18	15
Eggs/week	0	66	55	90	75	Marital status	Married	100	83.33	67	55.83
	>=1	54	45	30	25		Widow	20	16.67	53	44.17

**Table 2:** Parameter estimates and the Wald statistic value along with their *p* values. Odds ratios (ORs) and their corresponding 95% confidence intervals (CIs) are in the last two columns.

	Estimate	Wald Z	*p* value	OR	95% CI of OR
Age	0.09	2.54	0.01^*∗*^	1.10	(1.02, 1.18)
Locality (rural)	−1.10	−1.90	0.06	0.33	(0.11, 1.04)
BMI	−0.07	−1.59	0.11	0.93	(0.86, 1.02)
Literacy (literate)	−1.02	−1.52	0.13	0.36	(0.10, 1.34)
Awareness (yes)	−0.08	−0.08	0.94	0.92	(0.12, 7.22)
Symptoms (body pain)	−0.19	−0.30	0.77	0.83	(0.24, 2.84)
Fracture (yes)	1.27	1.98	0.047^*∗*^	3.55	(1.02, 12.38)
Fracture history (yes)	0.09	0.13	0.90	1.10	(0.28, 4.27)
Family history (yes)	3.59	2.91	<0.01^*∗*^	36.3	(3.23, 408.55)
Physical activities (yes)	−2.67	−4.45	<0.01^*∗*^	0.07	(0.02, 0.22)
Sun exposure (yes)	−0.32	−0.50	0.62	0.73	(0.21, 2.54)
Family size	0.21	2.19	0.03^*∗*^	1.24	(1.02, 1.49)
House (owned)	0.03	0.04	0.97	1.03	(0.19, 5.53)
Milk frequency per week (>=1)	0.19	0.35	0.73	1.21	(0.41, 3.54)
Meat (red)	−0.22	−0.26	0.80	0.80	(0.15, 4.41)
(Red + white)	0.73	0.88	0.38	2.07	(0.41, 10.49)
Eating meat per week (>=1)	−1.43	−2.48	0.01^*∗*^	0.24	(0.08, 0.74)
Eating eggs per week (>=1)	−0.64	−1.29	0.20	0.53	(0.20, 1.40)
Marital status (widow)	−0.38	−0.59	0.55	0.69	(0.20, 2.38)
No. of children	−0.21	−1.58	0.11	0.81	(0.63, 1.05)
Calcium supp. during pregnancy (yes)	0.72	0.89	0.37	2.04	(0.42, 9.92)
Delivery kind (normal)	−4.35	−2.27	0.02^*∗*^	0.01	(0.00, 0.55)
(Operate)	−2.85	−1.50	0.13	0.06	(0.00, 2.42)
Breastfeeding in past	1.96	1.61	0.11	7.12	(0.65, 77.73)
Currently breastfeeding	4.79	2.16	0.03^*∗*^	120.16	(1.56, 9277.49)
Menopausal status (abnormal)	2.11	2.87	<0.01^*∗*^	8.28	(1.95, 35.14)
Age at menarche	0.38	1.60	0.11	1.47	(0.92, 2.35)
Menstrual flow (normal)	−0.49	−0.64	0.52	0.61	(0.14, 2.74)
Menstrual cycle (>=28 days)	−0.15	−0.11	0.91	0.86	(0.05, 13.85)
Menstrual cycle repeat (regular)	−0.93	−0.59	0.55	0.40	(0.02, 8.39)
Cal. supplement >=1 time/week (yes)	0.30	0.41	0.68	1.35	(0.32, 5.75)
Appetite (normal)	−2.42	−4.02	<0.01^*∗*^	0.09	(0.03, 0.29)
Anticoagulants use (yes)	3.01	2.54	0.01^*∗*^	20.31	(1.98, 208.17)

^*∗*^Significant at the 5% level of significance.

## Data Availability

The dataset is available upon reasonable request from the corresponding author.
